# Stability Analysis of Geotechnical Landslide Based on GA-BP Neural Network Model

**DOI:** 10.1155/2022/3958985

**Published:** 2022-06-20

**Authors:** Jin Xu, Yanna Zhao

**Affiliations:** ^1^School of Civil Engineering, Xuchang University, Xuchang, Henan, China; ^2^Xuchang Jinke Resource Recycling Co., Ltd., Xuchang, Henan, China

## Abstract

Rock and soil landslides, a regular geological disaster in engineering construction, endanger national property and, in severe circumstances, result in a huge number of casualties. A set of methods for landslide stability analysis and prediction has been established, with the academic idea of “geological process mechanism analysis-quantitative evaluation” at its core, combined with detailed field investigation of geological hazards, forming a relatively complete technical route for research on landslide stability analysis. The work of this paper can be summarized as follows: (1) Introduce the research status of geotechnical landslide stability at home and abroad and the current development trend of neural network. (2) Through the collected sample database, take the training function and the number of hidden layer neurons as variables to optimize the BP neural network, and combine the optimized BP neural network with the genetic algorithm to construct the GA-BP neural network. (3) The stability coefficients of the BP neural network, the genetic algorithm based back propagation neural network (GA-BPNN), and the limit equilibrium technique are analyzed and compared. The findings imply that landslide stability can be assessed using neural networks. GA-BPNN is a viable alternative to back propagation neural network (BPNN). The algorithm is more accurate, has a faster convergence rate, and is more stable.

## 1. Introduction

Geotechnical landslide is a geological phenomenon of sliding of the slope rock and soil along the through shear plane caused by natural geological action and human engineering activities. Landslide instability and damage cause heavy losses and disasters. The EM-DAT catastrophe database estimates that 8,658 persons perished as a direct result of landslide activity throughout the globe during 1990 and 1991 [1]. “The Durham Fatal Landslide Database” (DFLD) database indicates that the death toll from landslide events between 1980 and 2000 was about 72,000 worldwide, or about 3,400 per year, a figure that is considered a significant underestimation of landslide hazard outcomes because the underreporting of small events (events with very low mortality rates) and events that occur in very remote areas keeps the count far below the actual number [2]. Landslide geological disasters are widely distributed in my country. According to statistics from the Ministry of Land and Resources, mountains in my country account for about 33% of the country's land area, plateaus account for 26%, and hills account for 10%. Usually people refer to mountains, hills, and relatively rugged plateaus as mountainous areas. Mountainous areas in my country account for more than two-thirds of the country's land area. One of the important reasons for the underdeveloped economy in the vast mountainous areas of our country is the poor topographic and geological conditions and the backward infrastructure, especially the transportation facilities. In order to fundamentally enhance the economic growth of these places, the state has been concentrating larger efforts in recent years and for a long time in the future to establish various infrastructures in these areas. There are many geological threats in large areas of mountainous areas. Various engineering constructions in the mountainous areas have more and more disturbances to the natural geology, coupled with natural factors such as climate change and seismic activity, resulting in frequent occurrence of geological disasters such as rock and soil landslides, hindering and limiting the occurrence of geological disasters. The development and construction of mountainous areas, especially in recent years, the rural highway network and the “eight vertical and eight horizontal” high-speed railway network, as the main artery of the national economy and the construction of major livelihood projects, are in full swing. Geotechnical landslides have been listed as one of the major geological disasters in my country, and key research has been carried out. The prediction and control of landslides has always been an important research direction in the field of geotechnical engineering. In order to better provide a basis for landslide prevention and control, it is necessary to deeply understand the mechanical mechanism and failure process of landslide instability and establish accurate stability evaluation standards to achieve scientific prevention and control and reduce and eliminate landslide disasters in engineering construction. Slope stability is a means of determining prevention measures and engineering quantities. The calculation of landslide safety factor is the basis for control design. Stability calculation is the core of slope stability analysis. Slope stability is a state that indicates whether the slope is safe or not and the degree of safety. The result of treatment should be to make the slope reach the safety standard state. Since slope rock and soil is a complex geological medium, it is difficult to obtain quantitative values accurately, so qualitative analysis based on geological statistics and experience should be combined with quantitative calculation. In the semiquantitative evaluation method, there is also the problem of artificially quantifying each factor index and determining the weight of the factor based on experience, which is difficult to truly reflect the actual situation. With the deepening of research, the phenomenon of interdisciplinary is becoming more and more common, so it has become a trend to study the stability of rock and soil landslides with new analytical methods. This paper mainly improves the traditional BP neural network based on the genetic algorithm, and applies the GA-BP neural network to the stability analysis of the landslide, aiming to seek a way to improve the prediction accuracy.

The paper organizations are as follows: Section 2 defines the related work.  Section 3 discusses the methods of the proposed concepts.  Section 4 discusses the analysis of experimental and discussions.  Section 5 concludes the article.

## 2. Related Work

The landslide mechanism is the physical and mechanical nature and laws of the whole process of the slope under certain geological structure conditions, from stable to unstable state under the action of various factors, and then to a new stable state or permanent instability. The concept of progressive failure of soil was first proposed by reference [3, 4]. The theory of stress differentiation and shear strength redistribution was used to explain the progressive failure, and it was pointed out that its essence was that the soil flowed from the initial strength state to the plastic flow, but only limited to the brittle clay range at that time. It is reference [5] that really applies the concept of progressive failure to slope analysis. By analyzing and studying the long-term stability of soil slopes, and analyzing the results of a large number of field direct shear tests, it is pointed out that the slope deformation changes from local to overall through failure. In the process, the research on the gradual development of the slope is developed on the basis of the traditional static research. After that, the gradual failure of the slope has made more development, and reference [6] studied the gradual failure mechanism of the slope from the perspective of failure criteria and stress-strain relationship according to the experimental study of soil strength. Reference [7] established a mechanical model of progressive failure of excavation slopes according to the strain softening characteristics of soil under fatigue load and considered that the discontinuity of the slope soil resulted in progressive failure. Reference [8] analyzes the development of cracks in the slope, applying various parameter combinations to represent the peak and residual shear strength conditions along the cracked and uncracked parts of the critical surface, and analyzes the progressive failure process. Reference [9, 10] established a calculation model for the gradual development of the slope from the toe to the top and explained the progressive failure mechanism from the perspective of probability analysis.

The stability analysis of rock and soil landslides has a research history of more than a century, and many scholars have achieved a series of achievements, forming the theoretical basis of slope analysis. There are currently a variety of methods for assessing the stability of geotechnical landslides, the most common of which are the geological analysis method, empirical analogy method, structural analysis method, limit equilibrium analysis method, numerical analysis method, and probability analysis method, the first three of which are qualitative analysis methods. However, the latter three are used more in the stability evaluation of rock and soil landslides. The limit equilibrium method regards the sliding body as a rigid body and analyzes its equilibrium state along the sliding surface. The commonly used methods include the Janbu method, the simplified Bishop method, the wedge body method, the transfer coefficient method, the Fellenius method, and the Sama method. These methods are all based on the limit equilibrium state, treat the rock and soil mass as a rigid body, and assume that the sliding zone as a whole reaches a critical state, which is far from reality in many cases and cannot reflect the real stress-strain relationship inside the rock and soil mass. A large number of studies have shown that the deformation and failure of slopes are a gradual process. Some scholars have extended the limit equilibrium method combined with the change of strength parameters and developed a system of gradual development research on the basis of traditional static research. Skempton put forward the concept of gradual failure of slope through the analysis and research of soil slope and developed the research of gradual development on the basis of traditional static research. Reference [11–13] considered the softening characteristics of soil strength parameters, and considered the mechanical mechanism and failure evolution process of the gradual development of the slope, and extended the limit equilibrium analysis method. The numerical analysis strength reduction method can calculate the stability of the slope in combination with the constitutive relationship of the rock and soil mass and can reflect the gradual failure process of the slope to a certain extent. The area where the shear strength is exceeded is the failure area. Reference [14] proposed the strength reduction method, which has been widely used in the numerical calculation of slope stability and is also developing continuously; the strength reduction method provides convenience for the calculation of various complex slopes; and the calculation amount and accuracy are guaranteed to a certain extent. The determination of the final result of the strength reduction method depends on the selection of the calculation termination conditions, that is, the choice of the instability criterion. Reference [15] takes the nonconvergence of a certain number of nonlinear iterative calculations as the instability criterion, and uses a large number of strength reduction methods and numerical calculations to demonstrate its feasibility [16]. Geological issues such as earthquakes, geophysical research, and geological hazard prevention and prediction have recently used neural network theory. In terms of geological disaster prevention and prediction, the application of domestic BP neural network can be roughly divided into three stages: understanding, development, and extension. The cognitive stage is the enlightenment period for the application of BP neural network to geological disasters. This period mainly provides a theoretical basis and is not used in practical engineering applications; in the development stage, geologists use BP neural network to solve landslides, land subsidence, and sand liquefaction. Extension of the BP neural network to a new study stage was made possible by geologists combining ideas and technology from other disciplines to create new research approaches [17]. Neural networks are projected to have a wide range of applications in multivariate analysis, parameter prediction, inversion, and factor sensitivity analysis in engineering geological issues. The danger elements impacting landslide stability were discovered after a thorough review of landslide stability assessment methodologies. Researchers have developed a novel approach for analyzing slope stress by combining discrete element computation with neural network prediction; an assessment model for town landslides' stability was developed by researchers using BP neural networks; and the forecast findings were in line with the actual circumstances. Abroad, a research group of scientists had insight into the importance of neural network information processing, and established a parallel and distributed processing (PDP) group in 1982 to explore parallel distributed processing technology, and three years later, the BP network learning algorithm was researched, and Minsky's multilayer network vision was realized [18]. Subsequently, reference [19] published three academic papers on the application of neural networks in distinguishing earthquakes from blasting. Reference [20] used a new method of GIS combined with artificial neural network model earlier to evaluate the landslide risk in the Boeun area of Korea. It can be seen from the above that in recent years, scholars at home and abroad have achieved many research results in engineering applications using BP neural network, especially the improvement of BP neural network combined with other disciplines. There are few studies related to prediction [21, 22].

## 3. Method

### 3.1. Construction of BP Neural Network Model

#### 3.1.1. Principle of BP Neural Network Algorithm

The following nodes make up the BP neural network: In other words, a BP neural network is used to teach the error back propagation method. The training process is divided into two stages. To determine your mistake, start by comparing your output value to a real-world value. The BP neural network has three layers: an input layer, a hidden layer, and an output layer. The training data enters the model through the input layer, which acts as a buffer for the data. It is up to the user to decide how many layers of the hidden layer they want, and the number of neurons in each layer is determined empirically by training and testing the model many times with different combinations of input data parameters. The input layer sends data to the hidden layer, which transforms it before passing it on to the output layer, which generates the forward-propagated data. The activation function of the output layer transforms data that has been passed from the hidden layer. The network performs the error back propagation process when the difference between the output result and the measured value is too large. The BP neural network gradient descent algorithm is used to correct each layer's weights and thresholds, and then, forward prediction is performed once more. End the training session now. The structure of the BPNN model is shown in Figure 1.

#### 3.1.2. BP Neural Network Parameter Selection

Many variables must be taken into account while creating a BP neural network model. The number of hidden layers, the number of neurons in the hidden layer, the starting weights, the activation function, the anticipated error, the learning rate, and the number of repetitions of learning, among other factors, are not precisely described.

Since there is just one hidden layer in the BP neural network, it is unknown how many layers it may have. However, this is plausible. If you have a three-layer BP neural network with only a single hidden layer, you can complete any nonlinear mapping, even if the nonlinear map goes from *n* to *m* dimensions. Despite the fact that the BP neural network's three layers can approximate any nonlinear mapping, there is a large difference between the output result and the actual value and a poor degree of accuracy in identification. Allowing for a greater number of hidden layers helps alleviate this drawback. A more complicated BPNN structure results from adding more hidden layers, since the weight training time for neuron connections across layers increases as more layers are added. Although adding more hidden layers improves the BP network's output accuracy, it is simpler to see and change the network training effect when there are more neurons in each layer. Therefore, increasing the number of hidden layers is the best method for reducing network training error.

The buried layer's neuron count is as follows: It is necessary to start with a small hidden layer to train and debug the neural network and then increase the number of neurons in the hidden layer until it performs to specifications. Increase the number of hidden layers if it does not work. It has been found that the process of adding hidden layer nodes is significantly easier than the process of adding hidden layers. If you have just one hidden layer in your neural network, you may use this method to figure out the number of nodes in the hidden layer's first layer.

(1) $$\begin{array}{c} \text{z}=\sqrt{q+p}+a, \end{array}$$

where *p* and *q* represent the number of nodes in the input layer and output layer, respectively, and *a* is a constant with a value range of (1, 0).

Activation function, learning rate, and expected error: The activation function is introduced into the BP neural network because the BP neural network model studies nonlinear problems, and the nonlinear function is introduced to increase nonlinear factors. When the activation function is introduced into the BP neural network, the network becomes more complex than before, thus improving the expressive ability of the network. However, there are certain restrictions when choosing the activation function; that is, the function must be derivable and continuous. There is an activation function for this paper's hidden layer that is called tansig, and its value range is between 1 and 1. Due to the fact that the normalized data in this study fall between -1 and 1, the output layer picks the purelin function, which is linear, in the MATLAB toolbox in order to expand the range of values for the output. For the tansig function, the following expression is appropriate:

(2) $$\begin{array}{c} f\left(x\right)=\frac{e^{x}-e^{-x}}{e^{x}+e^{-x}}, \end{array}$$

It can be obtained by simple operation. *f*(*x*) ∈ (−1, 1).

The mathematical equation for the first derivative of tansig is

(3) $$\begin{array}{c} f^{\text{'}}\left(x\right)=\frac{4}{{\left(e^{x}+e^{-x}\right)}^{2}}\tanh\left(x\right)=\mathrm{sech}{\left(x\right)}^{2}. \end{array}$$

A significant aspect in the BP neural network's success is its ability to adapt to changes in the model's weights throughout the training phase. If the learning rate is too high, the weights will change more often, resulting in a bigger change each time they are updated, and it is very likely that the optimal weights cannot be found or not easily found, and even the BP neural network will collapse. If the learning rate is too small, the time for each training weight update will be longer, reducing the convergence speed of the network. In practical applications, even if the learning rate is too small, it will affect the convergence speed of the network, but this method avoids the local optimal solution of the trained network, so a relatively small learning rate is often selected. The value range of the learning rate in the BPNN model is commonly found to be between 0.01 and 0.08. This article regularly trains the existing BP neural network-based geotechnical landslide prediction model with a learning rate of 0.01, and its performance is superior.

The expected error is very important for the BP neural network. It is an evaluation criterion for the excellent performance of the network model. In order to make the error of the BP neural network relatively small, the network structure and performance must be paid to a certain extent, increasing the number of hidden layers of the network or increasing the number of neurons in the hidden layer and consuming more training and learning time. In order to reduce the cost of the network, it is necessary to work on the expected error function. There are three kinds of error functions commonly used in BP neural network, and the following is the comparison of these three error functions. The error function commonly used in the BP network model is the formula *E*_*p*1_:

(4) $$\begin{array}{c} E_{p1}=\frac{1}{2}\overset{m}{\underset{j=1}{\sum }}{\left(t_{j}^{p}-y_{j}^{p}\right)}^{2}, \end{array}$$

where *m* is the number of neurons in the output layer; *p* is the number of training samples; *E*_*p*_ is the error of the *p* data of the training sample; *t*_*j*_^*p*^ is the true value; and *y*_*j*_^*p*^ is the output value.

Each time the BP neural network updates the weights, it will be affected by each sample. However, there are certain disadvantages in using this error function. It only considers the influence of the current sample on the weights, and does not consider the influences of other samples on the modified weights. Therefore, this error function will increase the training times of the BP neural network. The cumulative error *E*_*p*2_ is a global error function, which is defined as follows:

(5) $$\begin{array}{c} E_{p2}=\frac{1}{2}\overset{p}{\underset{p=1}{\sum }}\overset{m}{\underset{j=1}{\sum }}{\left(t_{j}^{p}-y_{j}^{p}\right)}^{2}=\overset{p}{\underset{p=1}{\sum }}E_{P1}, \end{array}$$

where *p* represents the data of p training samples; *E*_*p*2_ represents the expected error of the *p*-th training sample; MSE = 1/*mp*∑_*p*=1_^*p*^∑_*j*=1_^*m*^(*y*_*pj*_^,^ − *y*_*pj*_)^2^ represents the real value; *y*_*j*_^*p*^ represents the output value of each loop; and *m* represents the number of neurons in the output layer.

The role of the global error function is to reduce the global error of the system. If it is only used in a sample, it can only improve the global error accuracy of the sample, and cannot affect the error of each sample. In addition, it cannot be compared with the performance of other networks, because the error values are different for *m* and *p* in the formula on different networks; when *m* is constant, the larger *p* is, the larger the global error *E*_*p*2_ is; when *p* is changed, the larger *m* is, the larger the global error *E*_*p*2_ is. The mean square error function of the BP network is

(6) $$\begin{array}{c} \text{MSE}=\frac{1}{mp}\overset{p}{\underset{p=1}{\sum }}\overset{m}{\underset{j=1}{\sum }}{\left(y_{pj}^{,}-y_{pj}\right)}^{2}, \end{array}$$

where *m* represents the number of neuron nodes in the output layer; *p* represents the number of samples;  *y*_*pj*_^,^ represents the true value; and *y*_*pj*_ represents each training value.

#### 3.1.3. Limitations of BP Neural Networks

Although the BP neural network has many advantages and has been widely used and promoted, there are still some limitations in terms of its structure and performance. The problems mainly include the following aspects.

1. Since the learning rate of the network cannot be selected too large, the BP neural network training takes a long time
2. The BP neural network algorithm may generate a local minimum solution, because the gradient descent method may be used to obtain a local minimum solution when updating the weights. As an optimal solution, the BP neural network will make the weights converge to a certain value, but not necessarily the global optimal value
3. The hidden layer of the BP neural network finally uses several layers and the number of neurons in each layer. Only a few can make the network performance optimal, so far there is no clear formula or theory, and their numbers are determined by users using empirical formulas and repeated training. Therefore, the network performance is uncertain. If there are too many hidden layers and nodes in each layer, the system will be too complicated, and the training speed will be slow; otherwise, the target curve cannot be better fitted
4. The predicted value of BP neural network is unstable. For the same training samples and prediction samples, the results of each prediction are different

### 3.2. Establish a Neural Network Based on GA-BP

The BP neural network must be tuned because of its high volatility and proclivity for local optimal solutions. The genetic algorithm has global search ability and can improve the defects of the BP model, so this paper uses the genetic algorithm to optimize the BP neural network.

#### 3.2.1. Principle of Genetic Algorithm

The calculation process of genetic algorithm is mainly composed of coding, population initialization, fitness function evaluation, selection, crossover, mutation, and other modules. The following is a detailed discussion of each module of the genetic algorithm. For coding, before carrying out the genetic algorithm, an important work must be done to the solution of the problem, which is to encode it into a symbol that the genetic algorithm can operate, that is, the chromosome string. Binary, floating-point, mixed encoding, and other methods can be used to encode the issue solution, with floating-point encoding having the maximum accuracy. For the initial population, the convergence speed of the genetic algorithm and the accuracy of the feasible solution must be guaranteed, and the precondition is that the size of the population should be appropriate. If the size selection of the population is too large, individuals with low fitness will be eliminated early in the process of genetic algorithm optimization, the diversity of the population will be reduced prematurely, and the distribution of feasible solutions will become sparse. The number of local solutions is reduced, and the operation process will also converge prematurely, and the global optimal solution of the problem will be difficult to search. Similar to the requirements of BP neural network training samples, as the input of genetic algorithm, the distribution of individuals in the population and the characteristics of the population should be rich, and these two aspects must be considered when selecting input data. When the starting population's features are basic, the genetic algorithm is prone to premature and local convergence, which affects the accuracy of the algorithm optimization; thus, attempt to make the initial population's individual characters as rich as possible. However, a diverse distribution of population individuals can overcome the lack of a single individual trait, even if the population is scattered in the entire search space. Usually, the initial population size is selected in the range of 20 to 100. In the design of the fitness function, the fitness is an evaluation of the ability of the individual population to adapt to the natural environment. Similarly, the fitness function is also an evaluation of the adaptive ability of the individual in the evolutionary process of the genetic algorithm. History has proved that organisms follow a law in the process of evolution; that is, the driving force and purpose of evolution are to evolve in the direction of adapting to the current living conditions. Genetic algorithm is a simulation of biological evolution, and the convergence of objective function can be regarded as the goal and motivation of evolution. The genetic algorithm population solely executes optimization calculations using its own fitness function during evolution, and does not seek input from the outside environment. As a result, the fitness function used in the genetic algorithm has a significant impact on the algorithm's performance. Usually, the reciprocal of the objective function is used as the objective function of the genetic algorithm, as follows:

(7) $$\begin{array}{c} F\left(f\left(x\right)\right)=\frac{1}{1+c+f\left(x\right)}\;c\geq 0,c+f\left(x\right)\geq 0. \end{array}$$

For selection, selection is also called regeneration or replication. The step is that the individual string randomly selects a certain individual from the parent population as the genetic information of the offspring according to the size of the fitness to replicate. The selection operation has a decisive influence on the size of the crossover individual and its offspring. In crossover, the genetic information of the individual will be passed on to the next generation in the process of evolution, and at the same time, each generation of individuals will change themselves in order to adapt to the surrounding environment. Therefore, the crossover operator can be understood through this concept. The function of the crossover operator is to make the next generation appear new individuals that are different from the previous generation. After generations of evolution, the crossover operator continuously adds new individuals to the population to participate in the calculation and eliminates the old individuals. According to the rules of biological inheritance, the exchange of genetic information between two combined individuals will generate two completely new individuals, and this operation will be repeated between the new individuals until it converges to the optimal solution. In mutation, for biological evolution, the probability of mutation is very small. Similarly, in genetic algorithm, mutation operation will randomly replace the value of chromosome string, but the probability of this operation is very small. For example, a mutation operation replaces 0 s with 1 s on a string of binary chromosomes with a probability of 0.1. The influence of mutation operation on the optimization of genetic algorithm should not be underestimated. First, it can make the local search of the algorithm more thorough and increase the search accuracy and the speed of the local optimal solution, preventing premature convergence of the algorithm.

#### 3.2.2. Genetic Algorithm Framework Process

The genetic algorithm framework process is shown in Figure 2.

### 3.3. BP Neural Network Based on Genetic Algorithm

#### 3.3.1. The Basic Principle of GA-BP Algorithm

Due to the fact that its method can map the nonlinear connection between input and output of any issue, BP neural network is extensively employed in a broad range of industries. It is simple to slip into the local minimum value using the typical BP neural network, and it takes an extremely lengthy time to train. Consequently, it is vital to strengthen and optimize the BP network in order to overcome its weaknesses. Genetic algorithms are employed to optimize the BP network in this article, creating the GA-BP network model. To begin, the BP network uses the genetic algorithm to optimize its initial weights, and then, the BP network uses its own method to train weights and thresholds that match the error criteria based on those optimized starting weights. The research reveals that the GA-BP algorithm can improve the classic BP network model's existing flaws, and it is currently the most often used BP network optimization approach. The operation flow of the GA-BP algorithm is shown in Figure 3.

#### 3.3.2. Optimizing the GA-BP Algorithm

Whether the appropriate crossover operator *P*_*c*_ and mutation operator *P*_*m*_ can be selected has a great impact on the performance of the genetic algorithm. The reason why the genetic algorithm can generate new individuals, the crossover algorithm plays a decisive role. Through crossover operation, excellent traits can be combined advantageously and be inherited to the next generation with higher fitness value. Therefore, in order to obtain as many optimal individuals as possible, the value of *P*_*c*_ is usually relatively large. However, if the value of *P*_*c*_ is too large, excellent parent individuals will be included in the crossover category, which will destroy the preservation mechanism of excellent individuals and slow down the evolution rate. If the value of *P*_*c*_ is selected too small, the growth rate of new individuals in the population will become very slow, and the process of GA optimization will take too long. The usual range for the probability of *P*_*c*_ is (0.40, 0.99). Mutation *P*_*m*_ is one of the methods to avoid prematurity in the genetic algorithm, and it is also an important method for the population to generate new individuals. However, the probability of mutation in nature is very small. In order to improve the effect of mutation in the genetic algorithm, its value will be appropriately increased. However, if the value of *P*_*m*_ is too large, it loses its original significance in genetics; on the contrary, if the value of *P*_*m*_ is small, the precocious effect of mutation suppression genetic algorithm will no longer exist. *P*_*m*_ usually takes the value (0.0001, 0.1).

When the probability of crossover and mutation is determined, individuals with particularly high fitness may occupy all the positions of the population after several generations of inheritance, which makes the genetic algorithm converge prematurely, resulting in a high probability of obtaining a local minimum value. By analyzing this phenomenon, it is concluded that once the algorithm appears precocious, the fitness of many individuals in the population is very close. At this time, the fitness variance value of the population is very small, so the variance characteristics at this time can be used as a precocious evaluation index. For ease of calculation, let

(8) $$\begin{array}{c} E_{2}=\frac{1}{M}\overset{M}{\underset{i=1}{\sum }}\left|f_{i}-f_{\text{avg}}\right|, \end{array}$$

where *E*_2_ is less than a certain value, the genetic algorithm is judged to be premature, and then, the processing measures are taken. In this paper, the adaptive crossover and mutation algorithm are used to realize the connection between the probability change of the genetic operator and the individual fitness. The optimized algorithm is shown in the formula.

(9) $$\begin{array}{c} P_{ci}=P_{c}\times \left(1-\frac{f\left(x_{i}\right)}{\sum_{i=1}^{M}f\left(x_{i}\right)}\right), \end{array}$$

(10) $$\begin{array}{c} P_{mi}=P_{m}\times \left(1-\frac{f\left(x_{i}\right)}{\sum_{i=1}^{M}f\left(x_{i}\right)}\right), \end{array}$$

where *P*_*ci*_ and *P*_*mi*_ are the crossover and mutation probabilities of the *i*-th individual after optimization and *P*_*c*_ and *P*_*m*_ are the crossover and mutation probabilities of the original entire population, respectively. It can be calculated from the formula that when the population is precocious, the probability of individuals in the population being genetically manipulated will decrease as the fitness increases. Individuals with very small fitness will not be eliminated completely because their value is too small, which enriches the diversity of the population. The biggest difference from the traditional algorithm is that the probability of the improved crossover and mutation operator will change with the change of the individual itself. Therefore, the genetic algorithm optimized by using the genetic operator is more in line with the evolutionary rules of biology and has obvious inhibitory effect on the precocious phenomenon.

## 4. Experiments and Discussions

In the experimental and discussions section, we define the example analysis of geotechnical landslide, stability analysis of geotechnical landslides by BP neural network, stability analysis of GA-BP neural network, and comparison of two stability evaluation methods.

### 4.1. Example Analysis of Geotechnical Landslide

This paper takes a soil slope as an example. The slope aspect is about 12°, the rear elevation is more than 450 m, the slope is 26-29°, the elevation is between 423 and 456 m, and the terrain slope is about 23.5°. The landslide is the Quaternary loose gravel soil sliding and deforming along the top surface of the bedrock. The plane is approximately rectangular. The elevation of the Yellow Sea at the front edge is 425 m, and the elevation of the Yellow Sea at the trailing edge is 455 m. The width of the front and rear edges is about 80 m, and the middle is slightly wider. Calculated by the limit equilibrium algorithm, the stability coefficient of the landslide is 0.9956, and there is the possibility of overall slippage.

### 4.2. Stability Analysis of Geotechnical Landslides by BP Neural Network

Since the weights and thresholds of the neural network are randomly generated at the beginning of training, the results of each network training cannot be guaranteed to be consistent, and sometimes even large errors may occur; the trainlm function trains the neural network with high prediction accuracy for training samples, but not consistently high for detection samples. Therefore, in order to ensure the accuracy of the results, this paper makes 10 correlation predictions and then takes the average value. The results of the 10 operations are shown in Table 1.

The mean of the 10 sets of predicted values is 1.0243, the absolute error is 0.0287, and the relative error is 2.68%. As can be seen from the table, compared with the limit equilibrium method, the single maximum error of the BP neural network reaches 9.36%, but the average relative error is only 2.68%, and the prediction accuracy is relatively high.

### 4.3. Stability Analysis of GA-BP Neural Network

In order to reduce the random error of a single prediction, the GA-BP neural network also made 10 correlation predictions for the landslide and then took the average value. The operation results of its 10 predictions are shown in Table 2.

It can be seen from the table that the relative error of the predicted value of GA-BP neural network is between 0.10% and 3.86%, the error is small, and the stability is better. Its mean is 1.0078, the mean absolute error is 0.0122, and the mean relative error is 1.19%.

### 4.4. Comparison of Two Stability Evaluation Methods

The comparison between the absolute error and the relative error of the BP neural network and the GA-BP neural network stability evaluation method are shown in Figures 4 and 5.

It can be seen from the figure that the GA-BP neural network algorithm has faster convergence speed, higher accuracy, and better stability than the BP neural network algorithm. The average comparison of the relative errors between the two is shown in Figure 6.

## 5. Conclusion

This paper firstly introduces the basic knowledge of BPNN from the research history, application research, and other aspects; clarifies the origin, definition, characteristics, application, and existing defects of BPNN; and determines the BPNN in this research. Because of the neural network model structure, using neural networks in the analysis and prediction of rock and soil landslides has a strong theoretical basis. The genetic algorithm's premise is also examined, and a neural network based on GA-BP is built and optimized. The two stability evaluation methods and the traditional limit equilibrium method are used in the actual geotechnical measurement, and the results are as follows:

1. The GA-based BP neural network can effectively improve the convergence speed of the network, improve the solution space of the network, and overcome the problem that it is easy to fall into local minima, thereby improving the prediction accuracy of the network
2. The training process of the BP neural network is greatly affected by the initial weights and thresholds. In addition to the insufficient number of samples and incomplete input parameters, in practical applications, there is a large error in the single training result of the neural network, and the method of averaging multiple training results can effectively reduce this error, thereby improving the prediction accuracy
3. The results show that utilizing methods like the BPNN algorithm and the GA-BPNN algorithm, neural networks can be utilized to analyze the stability of the Baitupo landslide using the limit equilibrium approach. The GA-BPNN algorithm provides a quicker convergence time, more accuracy, better stability, and more dependable outputs compared to the BP neural network method
4. The landslide stability calculation shows that the landslide is in an understable state as a whole under natural working conditions, and there is a possibility of overall slippage
5. The sample database in this work selects 9 characteristics that affect landslide stability; however, the rock mass structure, geological structure, and other issues that are difficult to measure have not been taken into account, which will invariably have an impact on the results. Therefore, the scientific selection of influencing factors will be a reasonable quantification of nonquantitative factors and is a problem worthy of further study

## Figures and Tables

**Figure 1:** The structure of the BP neural network model.

**Figure 2:** Genetic algorithm framework process.

**Figure 3:** Operation flow of the GA-BP algorithm.

**Figure 4:** Comparison of absolute differences between the two methods.

**Figure 5:** Changes in relative difference between the two methods.

**Figure 6:** Average comparison of relative errors between the two.

**Table 1:** Prediction stability coefficient of BP neural network.

Serial number	Predictive value	Actual value	Absolute difference	Relatively poor
1	0.999	0.995	0.003	0.36%
2	0.998	0.995	0.003	0.33%
3	1.042	0.995	0.046	4.48%
4	1.098	0.995	0.102	9.36%
5	0.999	0.995	0.003	0.37%
6	0.999	0.995	0.004	0.40%
7	1.003	0.995	0.007	0.77%
8	1.006	0.995	0.011	1.12%
9	1.092	0.995	0.096	8.86%
10	1.003	0.995	0.007	0.75%

**Table 2:** Predicted stability coefficient of GA-BP neural network.

Serial number	Predictive value	Actual value	Absolute difference	Relatively poor
1	0.998	0.995	0.003	0.31%
2	1.023	0.995	0.027	2.69%
3	0.996	0.995	0.001	0.10%
4	1.001	0.995	0.005	0.55%
5	0.997	0.995	0.001	0.14%
6	1.026	0.995	0.030	2.99%
7	0.999	0.995	0.004	0.42%
8	1.001	0.995	0.005	0.56%
9	0.998	0.995	0.003	0.32%
10	1.035	0.995	0.040	3.86%

## Data Availability

The datasets used during the current study are available from the corresponding author on reasonable request.
